The article "Dumbbell shaped craniorbital cavernous hemangioma" was published in 2020. Journal: BMC Neurol.

# Dumbbell shaped craniorbital cavernous hemangioma

**DOI:** 10.1186/s12883-020-01734-z

**Published:** 2020-04-22

**Authors:** Xingping Qin, Farhana Akter, Lingxia Qin, Qiurong Xie, Yanfei Li, Hongkuan Yang, Xin Li, Guo Zhang, Songlin Wu, Renzhong Liu

**Affiliations:** 1 Department of Neurosurgery, Renmin Hospital of Wuhan University, 238 Jiefang Road, Wuhan, 430060 Hubei China; 2 Massachusetts General Hospital Cancer Center, Harvard Medical School, Boston, MA USA; 3 Department Molecular and Cellular Biology, Harvard University, Cambridge, MA USA; 4 Department of Neuroscience, University of Cambridge, Cambridge, UK; 5 Department of Neurology, Renmin Hospital of Wuhan University, Wuhan, China; 6 Department of Gynecology and Obstetrics, Renmin Hospital of Wuhan University, Wuhan, China; 7 Department of Orthopedics, The First Affiliated Hospital of Jinan University, Guangzhou, China; 8 Department of Neurosurgery, Tongji Hospital, Huazhong University of science and technology, Wuhan, China; 9 Department of Anesthesiology, Cancer Hospital of Hubei Province, Wuhan, China; 10 Department of Geriatrics, Renmin Hospital of Wuhan University, Wuhan, China

**Keywords:** Craniorbital tumor, Cavernous hemangioma, Orbit, Sphenoid

## Abstract

**Background:**

Cavernous hemangioma of the orbit is a benign tumor mostly located behind the eye globe, but it rarely spread into the brain, which is called cerebral cavernous malformation as well, the lesion in the brain is irregular and enlarged blood. Here we report one particular case of craniorbital cavernous hemangioma.

**Case presentation:**

A 53-year-old woman presented with exophthalmos of the right eye and reduced vision. Computerized tomographical (CT) scan showed osteolytic honeycomb radial changes of the outer plate of the skull. A magnetic resonance imaging (MRI) scan was performed to obtain further details. T1-weighted (T1W) imaging showed slightly low signal mixed with small patchy high signal. T2-weighted (T2W) imaging showed uneven high signal. There was obvious enhancement in the middle and no enhancement in the peripheral bars. A surgically manage was performed using a left frontotemporal approach, the tumor excised fully, and the histopathology results revealed a cavernous hemangioma. The patient recovered well in the follow-up. Post-operative CT scan identified the lesion was successfully resected, MRI scan also showed full resection and enhanced signal from the presence of fat.

**Conclusions:**

Craniorbital cavernous hemangioma is uncommon, however within the cranium, they can lead to numerous complications particularly if affecting the visual apparatus. it could be diagnosed by imaging, which CT scan shows osteolytic honeycomb radial changes of the outer plate of the skull, T1W imaging shows slightly low signal mixed with small patchy high signal, T2W imaging shows uneven high signal, it is obvious enhancement in the middle and no enhancement in the peripheral bars. The surgically manage is the ideally treatment when there are some symptoms.

The article "Dumbbell shaped craniorbital cavernous hemangioma" was published in 2020. Journal: BMC Neurol.

## Background

Cavernous hemangioma of the orbit is a benign tumor mostly located behind the eye globe, but it rarely spread into the brain, which is called cerebral cavernous malformation as well, the lesion in the brain is irregular and enlarged blood. Here we report one particular case of craniorbital cavernous hemangioma.

## Case presentation

A 53-year-old female presented to the Ophthalmology department with exophthalmos of the right eye and reduced vision. She was seen by the Ophthalmologist who noted reduced visual acuity in right eye (6/15) compared to the left eye (6/12). Visual field testing revealed a defect in the left upper quadrant of the right eye with enlargement of the blind spot. Both pupils were however of equal size, diameter of 2.5 mm and equally reactive to light. The patient was referred for a computerized tomographical (CT) scan, which showed osteolytic honeycomb radial changes of the outer plate of the skull, with external protrusion **(**Fig. 1**)**. The lesion originated from the right wing of the sphenoid bone, destroyed the outer plate and inner plate, extended to the ipsilateral middle cranial fossa and orbit, and showed a helioradial change. The trabecula of the bone was arranged from the center to the periphery in the shape of chrysanthemum petals. A magnetic resonance imaging (MRI) scan was performed to obtain further details. T1-weighted (T1W) imaging showed slightly low signal mixed with small patchy high signal. T2-weighted (T2W) imaging showed uneven high signal. There was obvious enhancement in the middle and no enhancement in the peripheral bars **(**Fig. 2**)**. Based on the destructive nature of this lesion, a decision was made to surgically manage this case. Using a left frontotemporal approach, the scalp and temporal muscle were dissected and the right frontotemporal bone flap was removed. The tumor tissue was found to be involving the right superior and lateral wall of the orbit and this was invading the dura matter. The tumor also extended to the right temporal bone and the right skull base. The tumor excised fully and the lesion was sent for histopathology. Free abdominal fat was taken to reconstruct the lateral wall of the orbit. The right frontal temporal bone flap was restored and fixed with cranial locking. Histopathology results revealed a cavernous hemangioma **(**Fig. 3**)**. A post-operative CT scan showed the lesion was successfully resected **(**Fig. 4**)**. A post-operative MRI scan also showed full resection and enhanced signal from the presence of fat **(**Fig. 5**)**. The patient was assessed immediately following the surgery by the operative surgeon. The exophthalmos in her right eye had resolved and the visual field was normal. Follow-up telephone consultation was performed 1 month after the surgery. The patient reported improved vision in the right eye compared to the left eye.

The article "Dumbbell shaped craniorbital cavernous hemangioma" was published in 2020. Journal: BMC Neurol.

**Fig. 1:** CT scan showing osteolytic honeycomb changes (arrow). The lesion originates from the right wing of the sphenoid bone, extends to the ipsilateral middle cranial fossa and orbit

**Fig. 2:** T1WI showing slightly low signal mixed with small patchy high signal. T2WI showing uneven high signal. There is enhancement in the center of the lesions but no enhancement in the periphery

**Fig. 3:** Resection approach for the tumor affecting the right temporal bone (A-D). Fully resected tumor (E). Histology revealed a cavernous hemangioma (F)

**Fig. 4:** Post-operative CT scan showing the lesion was successfully resected

**Fig. 5:** Post-operative MRI scan also showed full resection and enhanced signal from the presence of fat

## Discussion and conclusions

Cavernous hemangiomas of the skull are uncommon lesions and represent less than 1% of bone tumors [1]. Within the skull, they are most commonly located in the frontal bone and are very rarely found in the sphenoid or orbital rim, as seen in this case. Although they are considered benign, they can grow into surrounding tissue and cause localized damage. Hemangiomas are abnormal growth of small blood vessels, which can be classified according to their pathological types. The most common type is capillary hemangioma, which is characterized by a high density of small capillaries lined with a layer of endothelial cells. Cavernous hemangiomas are characterized by high density of large dilated blood vessels with distended ‘caverns’ filled with blood. Compound hemangiomas are a mixture of both capillary and cavernous. Hemangiomas can also be characterized according to their location and can be found in various organs such as the liver [2]. Hemangiomas can be further characterized as ‘congenital’, which is present at birth and is very rare or ‘infantile’, which is present shortly after birth and affects 4–5% of newborns [3]. Hemangiomas are often confused with vascular malformations, which consists of clusters of blood vessels that develop in particular blood vessels. They are usually more infiltrative than hemangiomas [2].

The molecular etiology of this hemangiomas is not well understood. A leading hypothesis is that endothelial cell proliferation and migration is key to the development of the disease [3]. However, the cause of this is not known. There is some evidence that there are mutations in genes regulating angiogenesis [4]. There is also evidence of increased expression of antigens associated with placental vessels in hemangioma [5]. The mechanisms underlying the spontaneous resolution of the disease is not well understood. A greater understanding of this process may also provide clues to the underlying pathobiology. There are many technical challenges of performing surgery on cavernous hemangiomas in the orbital region and therefore an understanding of the disease will help us to develop potential medical therapies, which may obviate the need to perform surgery.

The article "Dumbbell shaped craniorbital cavernous hemangioma" was published in 2020. Journal: BMC Neurol.

## Data Availability

The datasets supporting the conclusions of this article are included within the article.

## Abbreviations

CT: Computerized tomographical
MRI: Magnetic resonance imaging
T1W: T1-weighted
T2W: T2-weighted
